The article "An Entity Relationship Extraction Model Based on BERT-BLSTM-CRF for Food Safety Domain" was retracted in 2023. Reasons: unreliable results or conclusions; concerns about the data; concerns about the results or conclusions; concerns about the peer review.

# An Entity Relationship Extraction Model Based on BERT-BLSTM-CRF for Food Safety Domain

**DOI:** 10.1155/2022/7773259

**Published:** 2022-04-28

**Authors:** Qingchuan Zhang, Menghan Li, Wei Dong, Min Zuo, Siwei Wei, Shaoyi Song, Dongmei Ai

**Affiliations:** ^1^National Engineering Research Centre for Agri-Product Quality Traceability, Beijing Technology and Business University, Beijing 100048, China; ^2^School of E-Business and Logistics, Beijing Technology and Business University, Beijing 100048, China; ^3^Basic Experimental of Natural Science, University of Science and Technology Beijing, Beijing 100083, China

## Abstract

Dealing with food safety issues in time through online public opinion incidents can reduce the impact of incidents and protect human health effectively. Therefore, by the smart technology of extracting the entity relationship of public opinion events in the food field, the knowledge graph of the food safety field is constructed to discover the relationship between food safety issues. To solve the problem of multi-entity relationships in food safety incident sentences for few-shot learning, this paper adopts the pipeline-type extraction method. Entity relationship is extracted from Bidirectional Encoder Representation from Transformers (BERTs) joined Bidirectional Long Short-Term Memory (BLSTM), namely, the BERT-BLSTM network model. Based on the entity relationship types extracted from the BERT-BLSTM model and the introduction of Chinese character features, an entity pair extraction model based on the BERT-BLSTM-conditional random field (CRF) is established. In this paper, several common deep neural network models are compared with the BERT-BLSTM-CRF model with a food public opinion events dataset. Experimental results show that the precision of the entity relationship extraction model based on BERT-BLSTM-CRF is 3.29%∼23.25% higher than that of other models in the food public opinion events dataset, which verifies the validity and rationality of the model proposed in this paper.

## 1. Introduction

Food is the paramount necessity of the people and the material basis for human survival. Food safety is closely related to human health and has always been a concern of the society. With the development of the Internet and the wide application of computers, the Internet has penetrated into people's daily life. People have been accustomed to expressing their opinions on the Internet, so online public opinion has become an important channel to reflect social problems. Especially in recent years, food safety issues, such as dyed steamed buns, expired meat, poisoned bean sprouts, and other incidents have aroused high public concern. Some food safety incidents were not noticed until they were exposed on the Internet and finally solved. It can be seen that online public opinion is particularly important for the governance of food safety issues.

The article "An Entity Relationship Extraction Model Based on BERT-BLSTM-CRF for Food Safety Domain" was retracted in 2023. Reasons: unreliable results or conclusions; concerns about the data; concerns about the results or conclusions; concerns about the peer review.

With the progress of society and the awakening of people's health consciousness, people's demand for improving medical technology and enhancing health is more urgent. In the actual industrial development, China's smart healthcare is still in its infancy [1]. Smart health management is the application of artificial intelligence technology to specific scenarios of health management [2–6]. In terms of risk identification, through the acquisition of information and the use of artificial intelligence technology for analysis, we identify the risk of disease occurrence and provide risk reduction measures. In addition, virtual nurses can collect personal habit information about patients, such as eating habits, exercise cycles, and medication habits, and use artificial intelligence technology to analyze data and evaluate patients' overall status to help plan their daily life.

Therefore, by constructing the knowledge graph of public opinion events in the field of food safety, we can find food safety problems, prompt public opinion problems and give risk warnings, to make the connection between diseases clearer, and patients can receive treatment before complications occur, thus improving the health of patients. Extraction of public opinion events in the field of food safety is one of the important basic tasks in the construction of a knowledge graph in the field of food safety. Tao et al. [7] proposed crowdsourcing and machine learning approaches for extracting entities indicating potential food-borne outbreaks from social media using the dual-task BERTweet model. Mitra et al. [8] adopted a multiview deep neural network model for chemical-disease relation extraction from imbalanced datasets.

However, due to the diversity and universality of diseases caused by food safety incidents, there is a lack of a large number of available corpus in the field of food safety. Therefore, few-shot learning has become an effective method for information extraction. Gao et al. [9] proposed a multitask graph neural network based on few-shot learning for disease similarity measurement. Lu et al. [10] built a few-shot learning-based classifier by limiting training samples for food recognition. Sainz et al. [11] proposed a method of label verbalization and entailment for effective zero and few-shot relation extraction.

Extraction of public opinion events in the field of food safety is one of the important basic tasks in the construction of a knowledge graph in the food safety domain. The purpose is to extract semantic relationships between entities marked in sentences. Entity relationship extraction is mainly used to transform text unstructured data into structured data. The complexity of the entity relationship extraction task and the small sample of corpus lead to the difficulty to complete the task with few-shot learning. For the supervised deep learning model, the model is prone to underfitting due to the small sample corpus. On the other hand, the model is easy to fall into the local optimal solution, resulting in the poor actual effect of the model.

The article "An Entity Relationship Extraction Model Based on BERT-BLSTM-CRF for Food Safety Domain" was retracted in 2023. Reasons: unreliable results or conclusions; concerns about the data; concerns about the results or conclusions; concerns about the peer review.

This paper mainly studies an entity relationship extraction method based on BERT-BLSTM-CRF for the food safety domain. Based on few-shot learning, the whole model adopts the pipeline-type extraction method, which is divided into two tasks: entity relationship extraction and entity pair extraction. In the entity relationship extraction network model, the BLSTM network joined the BERT network trains on Chinese corpora, preprocessed to complete the entity relationship extraction task. In the entity pair extraction network model, to add feature information in the BLSTM network, this model puts the entity relationship extracted from the entity relationship extraction model to both ends of the character vector to reinforce the semantic features and obtain the radical feature to join the character vector. The model can not only handle entity overlap well but also effectively use the information of Chinese characteristics.

The rest of the article is organized as follows: Section 2 describes the related work.  Section 3 introduces the algorithm proposed in this paper.  Section 4 describes the environment we used to validate the algorithm as well as the experimental results and analysis. Finally, Section 5 summarizes this paper.

## 2. Related Work

The pipeline relationship extraction method [12–15] is popular in entity relationship extraction methods based on deep learning. In recent years, the problem of extracting multi-entity relationships in sentences has attracted the attention of researchers.

Bai et al. [16] proposed to extract local semantic features through word embedding and designed a new fragment attention mechanism based on CNN (convolutional neural network). Compared with the CNN model, the RNN (recurrent neural network) model can deal with distant patterns, so it is particularly suitable for learning relationships in longer contexts. Socher et al. [17] applied the matrix-recursive neural network model (MV⁃RNN) to natural language processing for the first time, which effectively solved the problem that the word vector model could not capture the constituent meaning of long phrases or sentences.

The article "An Entity Relationship Extraction Model Based on BERT-BLSTM-CRF for Food Safety Domain" was retracted in 2023. Reasons: unreliable results or conclusions; concerns about the data; concerns about the results or conclusions; concerns about the peer review.

The long short-term memory (LSTM) network model [18] has the same general framework as the RNN model, which has both forward pathways to transmit information and a self-feeding pathway to process information. However, LSTM allows each neural unit to forget or retain information. To some extent, the problem of vanishing or explosion gradient of RNN is solved. Zhang et al. [19] proposed a location-aware attention mechanism based on the LSTM sequence, which is combined with a kind of entity location-aware attention, to achieve better performance of relationship extraction. Huang et al. [20] proposed a new Chunk Graph LSTM network to learn the representation of solid blocks and infer the relationship between them. Chen and Hu [21] transformed the BLSTM-CRF deep learning model and improved sequence labeling rules.

In the latest research on natural language processing, the BERT model is a kind of network model which performs well in the present research stage. Instead of the traditional one-way language model or the method of shallow splicing of two one-way language models for pretraining, the algorithm adopts the new marked language model, which can generate deep two-way language representation and fine-tune specific downstream tasks [22]. At present, BERT has played an essential role in the research field of natural language processing, such as entity relationship extraction, text emotion analysis, and text classification [23]. Gao et al. [24] proposed a medical relationship extraction model based on BERT, which combined the whole sentence information obtained from the pretrained language model with the corresponding information of two medical entities to complete the relationship extraction task. Qiao et al. [25] proposed an agricultural entity relationship extraction model based on BERT-BLSTM-LSTM, which can effectively extract the relationship between agricultural entities.

In terms of the improvement of the model, Zhang et al. [26] proposed a new multi-label relationship extraction method based on a capsule network, which performed better than existing convolutional networks or cyclic networks in identifying highly overlapping relationships in a single sentence. Hang et al. [27] proposed an end-to-end neural network model for joint extraction of entity and overlap relations. Li et al. [28] proposed a new lightweight neural network framework to solve the problem of remote supervised relationship extraction. Xu et al. [29] proposed a new DocRE code-classifier-reconstruction model to extract document-level relationships and give more attention on the related entity pairs and path reconstruction. Sun and Wu [30] studied joint entity relationship extraction under remote supervision and developed a new adaptive algorithm that could deliver high-quality but heterogeneous entity relationship annotations robustly and consistently.

The article "An Entity Relationship Extraction Model Based on BERT-BLSTM-CRF for Food Safety Domain" was retracted in 2023. Reasons: unreliable results or conclusions; concerns about the data; concerns about the results or conclusions; concerns about the peer review.

However, in the papers mentioned above, most studies on entity relationship extraction are based on a large-scale corpus, while in the field of food safety, there is a lack of a large corpus. Moreover, in the literature given above, word vectors are used to represent semantic features of sentences, but unlike the foreign corpus, Chinese entities are usually grouped together in the form of characters. Furthermore, the radical feature of Chinese characters, which can reflect the semantics to some extent, has not been well used.

## 3. Methods

In Section 3.1, how to carry out manual annotation is introduced.  Section 3.2 describes how to construct the radical feature. In Section 3.3, the structure of the BERT-BLSTM-CRF model is introduced and the operating mechanism of the model is shown. In Section 3.4, this paper explains the detail of the extraction process of relationships of Chinese food public opinion event sentences.  Section 3.5 introduces the entities extraction model of food public opinion events sentences.

### 3.1. Manual Annotation

Firstly, entity relationship triples in sentences are extracted as shown in Figure 1, and then, sentences are processed into sequence labels as shown in Figure 2.

Sequence label in single relationship entity extraction consists of three parts, namely, entity boundary, entity relation, and entity role label. The entity boundary label is used by BIO to represent the location information of the element in the entity, where B indicates that the element is at the beginning of the entity, I indicates that the element is in the middle or end of the entity, and O indicates that the element is not an entity. Entity relationship labels in the corpus are shown in Table 1 in Section 4.1. The entity role tag represents the role of the entity in the triple, denoted by 1, 2, 1 for the subject and 2 for the object, for example, (metronidazole in edible duck egg exceeding bid, adverse reaction, nausea).

### 3.2. Construction of the Radical Feature

At first, Chinese sentences are divided into character units and then converted to radicals according to the correspondence defined in “Specification for Identifying Indexing Components of GB 13000.1 Chinese Characters Set,” as shown in Figure 3. For the problem that the simplified radicals are not defined in the word list of the pretrained model during the experiment, some of the simplified radicals are converted into normal Chinese characters by referring to the work of “Specification for Identifying Indexing Components of GB 13000.1 Chinese Characters Set” and the study by Chen and Hu [31].

The article "An Entity Relationship Extraction Model Based on BERT-BLSTM-CRF for Food Safety Domain" was retracted in 2023. Reasons: unreliable results or conclusions; concerns about the data; concerns about the results or conclusions; concerns about the peer review.

Formally, each Chinese character *f* in the sentence is added to *Cr*. And then, according to the rule of the radical decomposition, the radicals of the input sentence are generated and the radical *f*_*iv*_ of each character in the input sentence is added to *Cr*_*v*_.

(1) $$\begin{array}{c} Cr=\left[f_{1},f_{2},f_{3},\ldots ,f_{n}\right],\\ Cr_{v}=\left[f_{1v},f_{2v},f_{3v},\ldots ,f_{nv}\right]. \end{array}$$

Then, the vector representation *G*_*r*_ corresponding to the input *Cr*_*v*_ can be obtained through the one-hot method. Finally, we get the radical feature *G*_*r*_ of the input sentence.

(2) $$\begin{array}{c} G_{r}=\left[g_{v}^{1},g_{v}^{2},g_{v}^{3},\ldots ,g_{v}^{n}\right]\\ =\text{one }-\text{hot encoder}\left(Cr_{v}\right). \end{array}$$

### 3.3. Framework of the BERT-BLSTM-CRF Model

Figure 4 shows the structure of the BERT-BLSTM-CRF network model. The model is divided into left and right parts. Among them, the left half part of the figure shows the relationship extraction process of Chinese food public opinion events sentences. The right half part of the figure shows the extraction process of the entity pair of food public opinion events sentences.

In the relationship extraction model, as shown in the left half of Figure 4, after the sentence is put through the BERT, the character vector is obtained. Then, the BLSTM model which receives the character vector as input outputs the hidden layer vector, and finally, under the activation function of the sigmoid, the multirelationships can be obtained. The implementation details of the model are explained in Section 3.4.

In the entity pair extraction model, as shown in the right half of Figure 4, firstly, we obtain Chinese radicals in the field of Chinese food public opinion events and then get the Chinese radical feature representation by the one-hot method. In the BLSTM model, the character vector participates with the Chinese radical feature representation in the calculation of the intermediate hidden layer, and the entity relationships extracted by the model in left half part are added to the front and end of the hybrid character vector. After the BLSTM model outputs the hidden layer vector, the entity pairs are finally labeled under the function of the CRF method.  Section 3.5 will explain the specific implementation process of the model in detail.

### 3.4. Structure of the Relationship Extraction Model

The internal structure of the relationship extraction model is shown in Figure 5.

In order to strengthen the semantic features of Chinese, this paper chooses the way of character annotation, that is, the character is input as the basic unit.

The article "An Entity Relationship Extraction Model Based on BERT-BLSTM-CRF for Food Safety Domain" was retracted in 2023. Reasons: unreliable results or conclusions; concerns about the data; concerns about the results or conclusions; concerns about the peer review.

BERT is a language model trained by using a large number of unmarked texts in an unsupervised way. The encoder part based on the transformer carries out bidirectional coding. By constructing a marking language model, BERT can randomly cover or replace any word in a sentence, so that the model can predict the part that is randomly covered by the context and get the distributed context representation of the word. In addition, BERT performed the next sentence prediction task at the same time in the pretraining stage to make the model understand the relationship between the two sentences. Therefore, in order to enhance contextual semantic relevance, the BERT model is adopted in this paper. In the model of relational extraction, firstly, in the BERT, the characters loop through the Token Embedding layer, the Segment Embedding layer, and the Position Embedding layer. In the Token Embedding layer, [CLS] is put at the beginning of the sentence as the mark to be used for follow-on tasks to determine the kind of relationship.

The BLSTM receives the character vector generated by the BERT as input. In the BLSTM network, the character vector propagates forward and backward and the output layer outputs the final hidden layer vector. Finally, the sigmoid function is used to predict the multirelationship types, as shown in (3). The threshold value is trained by the neural network. When the value of the activation function is greater than the threshold value, it is judged to have a correlation and marked as 1; otherwise, it is judged to have no correlation and marked as 0. Finally, we get the relationship types.

(3) $$\begin{array}{c} \text{Sigmoid}=\frac{1}{1+e^{x}}. \end{array}$$

In this paper, we labeled seven types of relationships. We adopt seven bits to indicate whether there is a relevant correlation, where 1 represents correlation and 0 represents no correlation.

### 3.5. Structure of the Entity Extraction Model

The internal structure of the entity pair extraction model is shown in Figure 6.

To enhance the accuracy of entity recognition, entity semantics in statements need to be enforced. Firstly, the identified relationships are added to the hybrid vector to highlight the entities that need to be recognized. Secondly, Chinese characters have their own characteristics and radical features can represent a certain degree of Chinese meaning. Therefore, for the BLSTM model, the hybrid vector input is adopted.

At the input end of the BLSTM model, there are three kinds of inputs. The first one is the character vector generated by the BERT, and the second one is the Chinese radical feature representation. And then, one of the relationships extracted from the relational extraction model is constructed as the vector as long as the character vector which joins the Chinese radical feature and is added to the front and end of the hybrid character vector.

The article "An Entity Relationship Extraction Model Based on BERT-BLSTM-CRF for Food Safety Domain" was retracted in 2023. Reasons: unreliable results or conclusions; concerns about the data; concerns about the results or conclusions; concerns about the peer review.

The Chinese radical features of character have been obtained according to formula (2) as in Section 3.2. The character vectors are generated when Chinese characters pass through the BERT model, as shown in the following formula:

(4) $$\begin{array}{c} T=\left[t_{r}^{1},t_{r}^{2},t_{r}^{3},\ldots ,t_{r}^{N}\right]\\ =\text{BERT encoder}\left(Cr\right). \end{array}$$

Then, the character vectors are spliced with the radical features, as shown in the following formula:

(5) $$\begin{array}{c} R=\left[G_{r}☉T\right]. \end{array}$$

Next, we take one of the relations obtained in Section 3.4 and construct a relation vector *H*(*i*) as long as the splicing vector *R*, as shown in formula (6). Then, we divide the relation vectors into *t* parts, which are the kinds of relationship types, and the length of each part can be obtained by dividing the length of the splicing vectors by the kinds of relationship types. At last, we get the vector of the *i*^*th*^ relationship: the vector of the *i*^*th*^  segments are 1_*i*_^*k*^, and the vector of the other segments are 0_*i*_^*k*^.

(6) $$\begin{array}{c} H\left(i\right)=\left[0_{1}^{k},0_{2,}^{k}\ldots 1_{i}^{k},\ldots ,0_{t}^{k}\right]. \end{array}$$

Finally, the hybrid vector *K* is constructed by integrating *G*_*r*_,  *T*, and *H*(*i*), as shown in the following formula:

(7) $$\begin{array}{c} K=\left[\left[G_{r}☉T\right],H\left(i\right)\right]. \end{array}$$

After the sentence passes through the BERT and BLSTM models, only the relationship between the text sequence and tags can be obtained and the relationship between tags cannot be considered, so there will be many invalid predictive tags. Through the CRF layer, the obtained prediction tags are constrained to reduce the number of invalid prediction tags and obtain the global optimal tag sequence.

There are two types of scores in the CRF layer; one type is the tag probability *P* obtained through the BLSTM layer and the size of the matrix P is n^∗^m. *N* is the number of sentences, *m* is the type of tags, and *P*_*i*__*,j*_ is the probability of the label of the word in the sentence. And, the other type is the transition matrix *T*, and *T_i,j_* represents the transition probability from tag *i* to tag *j*. The sentence sequence *x = {x_1_, x_2_,..., x_n_}* corresponding to the tag sequence *y = {y_1_, y_2_,..., y_n_}* shown in the following equation:

(8) $$\begin{array}{c} s\left(x,y\right)=\sum_{i=1}^{n}\left(W_{yi-1,yi}+P_{i,yi}\right). \end{array}$$

The loss function of CRF consists of the real path score and the total score of all possible paths, as shown in the following equation:

(9) $$\begin{array}{c} \text{loss function}=\frac{e^{s\left(x,y\right)}}{\sum_{y\in \tilde{Y_{x}}}e^{s\left(x,\tilde{y}\right)}}. \end{array}$$

After the label probability and transfer probability in the CRF layer are obtained, the Viterbi algorithm is used to find the shortest path and the prediction label of each word in the sentence is obtained. The final hidden layer vector as the input passes through the conditional random field layer to mark whether the character is a subject or an object.

The article "An Entity Relationship Extraction Model Based on BERT-BLSTM-CRF for Food Safety Domain" was retracted in 2023. Reasons: unreliable results or conclusions; concerns about the data; concerns about the results or conclusions; concerns about the peer review.

The outputs of the BERT-BLSTM-CRF network model consist of four layers of output vectors. Two layers are the output vectors of subject labels in entity annotation, and the other two layers are the output vectors of object labels in entity annotation. Vector labels have no order and depend on input.

## 4. Results and Discussion

In Section 4, we introduce our experimental environment and parameter settings and compare the experimental results of entity relationship extraction with different models.

### 4.1. Experimental Dataset

In this paper, a field dataset (BBC) of food public opinion events in China is constructed as an experimental dataset. The corpus of the experimental dataset is from authoritative and professional websites in the field of food safety (such as China Quality News Network and Baidu Information about Food-Borne Diseases and Food Safety Events). In addition, another open (OP) dataset is used for comparison experiments to ensure the fairness of the experimental results. Among them, the corpus contains seven kinds of relationships. Table 1 lists the seven relationship types, as well as their names and abbreviations.

The experimental dataset and open-source dataset are divided into three parts: training set, validation set, and test set. The data volume size of each subset is shown in Table 2, and the details of the experimental dataset are given in Figure 7

In addition, to evaluate the effectiveness of BERT-BLSTM-CRF in different entity overlap scenarios, sentences in the BBC dataset are divided into normal (normal), entity pair overlap (EPO), and single entity overlap (SEO) according to different overlap types of relational triple, as shown in Figure 8. The normal class contains only one triple. In the SEO scene, only a single entity is shared at both ends of the relationship, such as the entity “excessive drug residues in turbot” in the sentence related to the entities Shanghai and Beijing. In the EPO scenario, the entities at both ends of the relationship are consistent, such as the entities in the triple < the crucian carps with enrofloxacin exceeding standard, Li Gang general store > overlapping.  Table 3 describes BBC experimental dataset division for different entity overlap scenarios.

The article "An Entity Relationship Extraction Model Based on BERT-BLSTM-CRF for Food Safety Domain" was retracted in 2023. Reasons: unreliable results or conclusions; concerns about the data; concerns about the results or conclusions; concerns about the peer review.

### 4.2. Evaluation Standard Setting

In this paper, three experimental results of precision, recall rate, and *F*1 value are used as performance measurement standards. The calculation formulas are shown as follows:

(10) $$\begin{array}{c} P_{i}=\frac{TP_{i}}{TP_{i}+FP_{i}}. \end{array}$$

In precision calculation formula (10), the precision as shown previously is referred to as *P*. *TP*_*i*_ represents the number of positive classes predicted by the model correctly and *FP*_*i*_ represents the number of positive classes predicted by the model from negative classes.

(11) $$\begin{array}{c} R_{i}=\frac{TP_{i}}{TP_{i}+FN_{i}}. \end{array}$$

In recall calculation formula (11), the recall as shown previously is referred to as *R*. *TP*_*i*_ is as the same as the above-mentioned formula and *FN*_*i*_ represents the number of negative classes predicted by the model from positive classes.

(12) $$\begin{array}{c} F1=\frac{P*R*2}{P+R}. \end{array}$$

The dataset of BBC-DATA constructed in this paper is a balanced dataset. Since precision and recall are a pair of contradictory indicators, to evaluate the performance of the classifier better, the harmonic mean *F*1 score of precision and recall rate is adopted as the evaluation standard to evaluate the comprehensive performance of the model.

### 4.3. Experimental Parameter Settings

In terms of experimental parameter setting, the main parameter information of the model in this experiment is determined by training the model and adjusting the parameters constantly. Among them, the BERT model's hidden layer has 12 layers, the vector has 768 dimensions, and the BLSTM model's hidden layer has 256 dimensions. An open-source deep learning framework based on PyTorch (https://pytorch.org/) is used to construct a deep learning model for experimental platform development. The main parameter information of the model proposed in the experiment is shown in Table 4 The hyperparameters in the experiment are determined by experiment and corpus, in which the dimension of character embedding is based on the experiment, the pad size is based on the maximum length of the sentence, and the learning rate is adjusted by the experiment.

### 4.4. Experimental Results and Analysis

In this paper, the proposed BERT-BLSTM-CRF model is experimentally compared with several other classical neural network models and models with an added attention mechanism. As shown in Table 5, the BERT-BLSTM-ATT model was proposed in [15]. In this experiment, seven annotated relationships are selected to conduct comparative experiments on independently constructed datasets and open datasets. The experimental results of each model relationship identification, including precision, recall rate, and *F*1 score, are shown in Table 5.

The article "An Entity Relationship Extraction Model Based on BERT-BLSTM-CRF for Food Safety Domain" was retracted in 2023. Reasons: unreliable results or conclusions; concerns about the data; concerns about the results or conclusions; concerns about the peer review.

The experimental results in Table 5 show that in the food public opinion events corpus and the open-source dataset, the precision of the BLSTM-ATT model is better than that of the CNN-ATT model, but CNN-ATT is better than BLSTM-ATT in recall rate and the overall effect of BLSTM-ATT is better. It can be seen from experiments 1, 2, 3, and 4 that the extraction precision of the neural network model is greatly improved after the attention mechanism is added. In the latest research on relation extraction, BERT learned a better text feature through the deep learning model, which further improved the overall performance of the model. In experiment 4, the BERT model is introduced into the BLSTM-ATT model and its accuracy is significantly higher than in the original model, which further verifies this point. The BERT-BLSTM-CRF model with no attention mechanism proposed in this paper adopts the BLSTM network model and the BERT network model. It is shown that the relational extraction precision and recall rate of the BERT-BLSTM-CRF model adopted in this paper have been greatly improved in the small sample dataset of the food public opinion events corpus and open-source dataset of large-scale corpus. Furthermore, its *F*1 value is the best.

After extracting the relationship, to test the effectiveness of entity pair extraction of the model proposed in this paper in the field of entity recognition of food public opinion events in China, this paper uses the same neural network model mentioned above for comparative experiments. The specific experimental results are shown in Table 6.

After extracting multiple relationships, the BLSTM model is only used to extract entity pairs. Experiments showed that the BERT-BLSTM-CRF model performs better with datasets. BERT-BLSTM-CRF offers significant improvements in precision and recall rate, and F1 also offers the best performance. For entity recognition, the BERT-BLSTM-CRF network model makes use of extracted relationships and Chinese radical features to reinforce the semantics of entities in sentences and enhance the entity recognition ability of the whole network. It is worth noting that the BERT-BLSTM-CRF network model constructed in this paper has good performance in both precision and recall rate, because not only BLSTM in the model can deal with the long-distance dependency problem in time series modelling but also BERT can introduce a deep learning model to learn a better text feature.

The article "An Entity Relationship Extraction Model Based on BERT-BLSTM-CRF for Food Safety Domain" was retracted in 2023. Reasons: unreliable results or conclusions; concerns about the data; concerns about the results or conclusions; concerns about the peer review.

This paper also verifies the BERT-BLSTM-CRF model's ability to extract relational triples from sentences with different numbers of triples. The sentences in the dataset are divided into five categories according to the number of different triples in the sentence, and the number of triples in the sentences is denoted by *N*.  Figure 9 shows the results of each model with different numbers of triples. It is obvious that the performance of the baseline model, including precision, recall rate, and *F*1 score, decreases with the increase of the number of triples included in sentences. Here, precision, recall rate, and *F*1 score are calculated according to the number of correctly extracted triples. Although the BERT-BLSTM-CRF model also showed a downward trend, it achieved excellent performance in all five classes. Compared with the baseline models, the model in this paper is least affected by the increasing complexity of input sentences, which also proves that the BERT-BLSTM-CRF model has achieved considerable improvement. At the same time, the biggest improvement of the BERT-BLSTM-CRF model in the BBC dataset comes from the most difficult cases (*N* ≥ 5), which also indicates that the model in this paper is more suitable for complex scenarios than the baseline model.

To further investigate the ability of the BERT-BLSTM-CRF model to extract overlapping triples, experiments are carried out on different types of sentences and the performance is compared with that of the baseline model.  Figure 10 shows the detailed experimental results of three different sentence types. It can be seen that the performance of all models in normal, EPO, and SEO sentence classification shows a decreasing trend, which also reflects that with the increase in sentence complexity, the difficulty of extracting relational triples from these three overlapping patterns is increasing. In other words, among the three overlapping cases, the normal class is the easiest sentence form to extract, while the EPO class and SEO class are relatively difficult cases to extract. In contrast, the BERT-BLSTM-CRF model achieves better performance in the extraction of three sentence types. It is worth noting that the experimental effect of the EPO scenario is better than the effect of the SEO scenario on the BERT-BLSTM-CRF model. The reason is that the model adopts the pipeline-type extraction method, which extracts the relationship first and then the entity. Therefore, the improvement of the relationship extraction can improve the extraction effect of the entity to a certain extent and thus improve the extraction effect of the triplet.

The article "An Entity Relationship Extraction Model Based on BERT-BLSTM-CRF for Food Safety Domain" was retracted in 2023. Reasons: unreliable results or conclusions; concerns about the data; concerns about the results or conclusions; concerns about the peer review.

The decreasing trend of the loss function of the BERT-BLSTM-CRF model proposed in this paper is shown in Figure 11. At the beginning of model training, many parameters of BERT have just been initialized and have not been adjusted for many iterations, so BERT does not have a good effect and the loss function has a large value. However, as the number of iterations of model training increases and the parameters are adjusted to a better state, the performance of the BERT-BLSTM-CRF network is gradually improved and the value of the loss function is gradually reduced.

## 5. Conclusions

This paper proposes a BERT-BLSTM-CRF relationship entity extraction model based on the corpus of food public opinion events in China. This model adopts the BLSTM model, BERT model, and CRF algorithm and performs training on a small sample corpus to complete the entity relation extraction task of transforming unstructured data into structured data. By constructing the BERT network model and the BLSTM network model, we predict the multirelationship in one sentence. Then, the splicing character vector is constructed by the character vector generated by the BERT joining the Chinese radical feature in the field of food safety events. One of the multirelationships is put on the front and the end of the splicing character vector of the sentence. Finally, CRF is used to mark the entity pair. The comparison experiment results show that the model proposed in this paper performs better than the previous deep neural network model.

The BERT-BLSTM-CRF model can solve the problem of entity relationship in the field of food safety by few-shot learning, which provides the basis for smart healthcare and security guarantees for human health. The model in this paper can not only have a good performance for multirelationship and multi-entity extraction problems but also handle entity overlap well. However, it has a limit for the number of entity pairs. Therefore, we will further explore how to solve more entity problems in Chinese entity relation extraction, such as the improvement of annotation methods, and transfer the proposed method to other application fields such as agricultural image recognition, greenhouse environmental time-series prediction, food safety risk assessment, and image recognition [32–40].

## Figures and Tables

**Figure 1:** Manual annotation instance.

**Figure 2:** Sequence annotation instance.

**Figure 3:** The radical feature construction.

**Figure 4:** Structure diagram of the BERT-BLSTM-CRF model.

**Figure 5:** The framework of the relationship extraction model.

**Figure 6:** Entity extraction model structure diagram.

The article "An Entity Relationship Extraction Model Based on BERT-BLSTM-CRF for Food Safety Domain" was retracted in 2023. Reasons: unreliable results or conclusions; concerns about the data; concerns about the results or conclusions; concerns about the peer review.

**Figure 7:** Details of the BBC experimental dataset.

**Figure 8:** Different overlap types of relational triple.

**Figure 9:** Precision, recall rate, and *F*1 scores for different number of triples.

**Figure 10:** Precision, recall rate, and *F*1 scores of relational triples in different overlapping patterns.

**Figure 11:** The loss function trending graph.

**Table 1:** Definition of relationships for the BBC dataset.

ID	Relation name	Abbreviations
1	Time	TI
2	Scene	SC
3	Name of food	NF
4	Food contaminant	FC
5	Adverse reaction	AR
6	Manufacturer	MF
7	Inspection body	IB

**Table 2:** Experimental dataset.

Dataset	Training	Validation	Test	Label
BBC-DATA	1500	300	400	7
OP-DATA	180000	50000	50000	35

**Table 3:** BBC experimental dataset division for different entity overlap scenarios.

Dataset	Training	Validation	Test
Normal	573	96	143
EPO	281	35	79
SEO	646	169	178

**Table 4:** Experimental parameter setting.

Model	Parameters	Value
BERT	Layer	12
	Dimensions	768
	Learning rate	5*e* − 5
	Pad size	128
	Function	Tan*h*

BLSTM	Layer	2-Layer
	Dimensions	256
	Learning rate	1*e* − 3
	Pad size	128
	Function	ReLu Tan*h*

**Table 5:** Experimental results of relationship extraction.

Model	BBC-DATA			OP-DATA		
	*P*%	*R*%	*F*1%	*P*%	*R*%	*F*1%
CNN	68.77	69.22	68.99	66.37	67.65	67.00
CNN-ATT	72.37	73.33	72.39	71.65	73.25	72.44
BLSTM-ATT	77.37	71.33	74.23	75.25	70.37	72.72
BERT-BLSTM-ATT	86.65	86.25	87.44	84.22	83.37	83.79
BERT-BLSTM-CRF	95.48	95.12	95.30	96.15	95.82	95.98

**Table 6:** Experimental results of entity extraction.

Model	BBC-DATA			OP-DATA		
	*P*%	*R*%	*F*1%	*P*%	*R*%	*F*1%
CNN	69.23	69.72	69.47	66.37	67.65	67.00
CNN-ATT	72.89	73.88	73.38	71.65	73.25	72.44
BLSTM-ATT	77.85	71.87	74.74	75.25	70.37	72.72
BERT-BLSTM-ATT	89.19	86.78	87.97	84.22	83.37	83.79
BERT-BLSTM-CRF	92.48	91.82	92.15	93.15	92.42	92.78

## Data Availability

The datasets used in this paper are available from the corresponding author upon request.
